# Tunicamycin-Induced Endoplasmic Reticulum Stress Promotes Breast Cancer Cell MDA-MB-231 Apoptosis through Inhibiting Wnt/*β*-Catenin Signaling Pathway

**DOI:** 10.1155/2021/6394514

**Published:** 2021-07-15

**Authors:** Zhongsheng You, Linkang He, Nianlong Yan

**Affiliations:** ^1^Department of Biochemistry and Molecular Biology, College of Basic Medical Science, Nanchang University, Nanchang, Jiangxi 330006, China; ^2^Queen Mary University of London, Nanchang University, Nanchang, Jiangxi 330006, China

## Abstract

Triple negative breast cancer (TNBC) has significantly threatened human health. Many aspects of TNBC are closely related to Wnt/*β*-catenin pathway, and cell apoptosis induced by endoplasmic reticulum stress (ER stress) in TNBC may act as a potential target of non-chemotherapy treatment. However, how ER stress interacts with this pathway in TNBC has not yet been understood. Here, the tunicamycin and LiCl have been applied to MDA-MB-231. The related proteins' expression was measured by western blotting. Moreover, acridine orange/ethidium bromide (AO/EB) staining was applied to test the apoptosis degree of the cells, and cell viability was tested by MTT experiment. Then, we found the ER stress and apoptosis degree of MDA-MB-231 were induced after treatment with tunicamycin. Besides, tunicamycin dose dependently inhibited both Wnt/*β*-catenin pathway and cells viability. Licl, an activator of Wnt/*β*-catenin signaling pathway, could significantly inhibit cell apoptosis. In conclusion, our study found that the activation of ER stress could promote the MDA-MB-231 apoptosis by repressing Wnt/*β*-catenin pathway, which provides some promising prospects and basic mechanism to the further research.

## 1. Introduction

All over the world, breast cancer has become the most severe cancer in women [1, 2]. In addition, triple-negative breast cancer (TNBC), with the worst prognosis as it lacks estrogen receptors (ERs), human epidermal growth factor receptor 2 (HER2), and progesterone receptors (PRs), has the highest mortality compared to the other types of breast cancer [3, 4]. A lot of research has investigated the relationship between breast cancer and Wnt/*β*-catenin signaling pathway [5, 6], which states that the initiation of Wnt/*β*-catenin pathway triggers the poor prognosis for TNBC [7]. The reduced phosphorylation of *β*-catenin induces the *β*-catenin deposition in nucleus and facilitates downstream genes' expression, for instance, cyclin D1 and c-Myc, which promotes the metastasis and drug resistance of cells [8, 9].

Endoplasmic reticulum (ER) stress has a certain toxic effect on cells, and it can be activated by a variety of stimuli, such as large amount of unfolded protein accumulation in cells, disorder of redox response, and calcium regulation disorder [10, 11]. Excessive misfolding protein could surpass the regulation ability of cells which are assisted by protein chaperones such as GRP78 and ultimately result in cell death by apoptosis [12]. Zhong et al. investigated the mechanism that promoting ER stress could cause the autophagy, apoptosis, and chemosensitivity of breast cancer through the PI3K/AKT/mTOR signaling pathway [13]. The relationship between ER stress, unfolded protein response, and apoptosis provides novel molecular targets for breast cancer treatment [14, 15]. Moreover, tunicamycin, which is a mixture of antibiotics, is used as an experimental tool to induce unfolded protein response, because it can block N-linked glycosylation and arrest the cell cycle in the G1 phase [16]. Therefore, the tunicamycin was used as an inducer of ER stress in our research.

The studies mentioned above explain the significance of Wnt/*β*-catenin pathway for TNBC. Furthermore, ER stress, as a regulator in the initiation process, is involved in cancer cell apoptosis through multiple pathways. Nevertheless, whether ER stress can reverse the apoptosis of TNBC through the inhibition of this pathway remains unknown. So, we intended to reveal the association between the injury of MDA-MB-231 induced by tunicamycin and Wnt/*β*-catenin pathway.

## 2. Materials and Methods

### 2.1. Cell Lines and Cell Cultures

The breast cancer cells MDA-MB-231 were acquired from the Chinese Academy of sciences (The Cell Bank of Type Culture Collection, Shanghai, China), and Dulbecco's Modified Eagle Medium (DMEM) obtained from the Healthcare Life Sciences (HLS) were used to culture MDA-MB-231 cells (HyClone; Logan, UT, USA); DMEM was included 10% fetal bovine serum (FBS) which acquired from the Biological Products Technology of Tianjin Haoyang. The culture condition of these cells was in the 5% CO_2_ and at 37°C.

### 2.2. MTT Assay Measures Cell Viability

The cells were transferred onto 96-well plates, and there are 5000 cells in each well. 20 *μ*L MTT was applied, respectively, to the well 24 hours after treatment. After four hours of incubation, the medium in each well was removed and purple precipitation was dissolved with 180 *μ*l DMSO. Finally, the spectrophotometer was used to detect the optical density at a 450 nm wavelength.

### 2.3. Western Blotting Analysis

RIPA lysate is added to the collected cells and is thoroughly mixed to obtain the proteins. The proteins of each group were electrophoresed on 10% gel in equal quantities. Then, the PVDF membrane was used to receive all the proteins and the PVDF membrane was sealed by 5% skim milk. The primary antibodies were applied subsequently onto the PVDF membrane to detect the expression of apoptosis-associated proteins Bcl-2 (cat. no. 60178-1-lg; dilution, 1 : 10000; ProteinTech Group, Inc.) and Bax (cat. no. 50599-2-lg; dilution, 1 : 12000; ProteinTech Group, Inc.), Wnt/*β*-catenin pathway-associated proteins *β*-catenin (cat. no. 51067-2-AP; dilution, 1 : 4000; ProteinTech Group, Inc.) and phosphorylated *β*-catenin (cat. no. DF-2989; dilution, 1 : 2000; Affinity Biosciences), key molecules of ER stress GRP78 (cat. no. 66574-1-lg; dilution, 1 : 50000; ProteinTech Group, Inc.) and CHOP (cat. no. WL00880; dilution, 1 : 1000; Wanleibio Co., Ltd), and regulatory gene c-Myc (cat. no. WL01781; dilution, 1 : 1000; Wanleibio Co., Ltd) and GAPDH (cat. no. HRP-60004; dilution, 1 : 50000; ProteinTech Group, Inc.). After TBST washing, the primary antibody which combines with the protein functioned as a platform to receive the combination of the secondary antibody. Lastly, an enhanced chemiluminogenic enhancer reagent was bought from Beijing Kangwei Century Biotech (cat. no. CW0049M). An autoradiography system bought from Bio-Rad Laboratories (Chemiluminescence Imaging System; version 5.1) was used to detect the blot. Every result was obtained by repeating the experiment three times and measured by Image Lab (Bio-Rad Laboratories; version 5.1).

### 2.4. Acridine Orange and Ethidium Bromide Staining (AO/EB Staining)

In 24-well plates, cells with treatment were cultured in 24-well plates for 24 hours. After the medium was removed from each well, 500 *μ*l of TBST containing AO/EB at 1 : 1 ratio was added to each well. After 5 minutes, the medium of AO/EB and TBST was discarded and the plates were washed using TBST three times. Finally, a fluorescence microscope was used to detect the fluorescence intensity.

### 2.5. Statistical Analysis

GraphPad Prism 6.0 was used to analyse all results. One-way analysis of variance (ANOVA) was selected to analyse the differences among each group, experiments were repeated three times; *P* < 0.05 represents statistical significance.

## 3. Results

### 3.1. Tunicamycin Effectively Inhibited MDA-MB-231 Cell Viability and the Wnt/*β*-Catenin Pathway

To detect the influence of tunicamycin for MDA-MB-231, the various concentration of drug was used to treat cells to determine their optimal concentration. The results showed that the ER stress key molecules GRP78 and CHOP increased as the dose of tunicamycin increased from nil to 2 *μ*mol/L (Figure 1(a)). At same time, tunicamycin promoted the Bax and phospho-*β*-catenin expression; meanwhile, it inhibited the expression of Bcl-2 and *β*-catenin dose dependently (Figures 1(b) and 1(c)). When tunicamycin dose was higher than 1 *μ*mol/L, the drug decreased the Bax and phospho-*β*-catenin expression but increased the expression of *β*-catenin and Bcl-2. To further evaluate the results of this experiment, the viability of cell was measured by MTT. The cell viability increased as the drug dose increased and reached a maximum at a dose of 1 *μ*mol/L of tunicamycin (Figure 1(d)). Therefore, the function of tunicamycin on cells and its suppressive effect in Wnt/*β*-catenin pathway is obvious when the concentration is at 1 *μ*mol/L; thus, in further experiments, this concentration was selected. In summary, this initially indicated that tunicamycin could repress the Wnt/*β*-catenin pathway and cell proliferation.

### 3.2. ER Stress Inhibits the Wnt/*β*-Catenin Signaling Pathway

LiCl can activate Wnt/*β*-catenin pathway, and Tunicamycin is an ER stress stimulator. In Figure 2(a), after treatment of tunicamycin and LiCl, *β*-catenin protein expression decreased by 48% and increased by 24%; however, phospho-*β*-catenin levels had a 200% increase and had a 51% decrease, respectively. In Figure 2(b), as for ER stress-related molecules, GRP78 protein expression decreased by 58% and increased by 45%, and CHOP increased by 135% and decreased by 38%. Therefore, these data indicated that tunicamycin inhibited the Wnt/*β*-catenin pathway; in summary, ER stress can affect this signaling pathway.

### 3.3. Tunicamycin Inhibits the Viability of MDA-MB-231 Cells via the Wnt/*β*-Catenin Pathway

It has been suggested that tunicamycin-activated ER stress can influence the Wnt pathway and increase the apoptosis rate in MDA-MB-231 cells. To further elucidate this potential mechanism, the expression of apoptosis-associated protein Bcl-2 and Bax was analysed (Figure 3(a)). The expression of Bax protein in the Tun and Li groups increased by 54% and decreased by 51% compared to the C group. Moreover, the level of Bcl-2 in the Tun and Li groups were reduced by 35% and increased by 172%. Compared with the Tun group, the Bax level in Tun + Li group was lower. However, the Bax level is lower in the Li group.

Next, we evaluated the effect of tunicamycin on ER stress on cell apoptosis. In Figure 3(b), AO/EB staining was used to measure apoptosis. Apoptosis of the cell in the Tun group enhanced by 47% compared to the C group and, in the Li group, by 18%, whereas compared with the Tun group or Li group, the apoptosis rates in the Tun + Li group were lower or higher. To sum up, these results demonstrated that tunicamycin-induced ER stress inhibited cancer cell growth through inducing the apoptosis of MDA-MB-231 cells.

To further elucidate the mechanism in the Wnt/*β*-Catenin pathway, our study next examined the c-Myc expression. The results indicated that, in MDA-MB-231 cells, the c-Myc expression levels were decreased after the treatment of tunicamycin (Figure 3(c)). Taken together, it was confirmed that the ER stress could shut the Wnt pathway, triggered the nuclear *β*-catenin decreasing, concurrently affected the downstream gene c-Myc transcription, and ultimately promoted MDA-MB-231 cell apoptosis.

## 4. Discussion

In ER stress, GRP78 and CHOP are essential in the regulation of unfolded protein response and ER stress [17, 18]. The results of GRP78 and CHOP from Figure 1(a) verified the ER stress was activated and confirmed that the ER stress degree in cells aggravated along with the increasing concentration of tunicamycin in MDA-MB-231 cells. Furthermore, Figure 1(b) reveals that the ER stress is affected by Wnt pathway. Concurrently, many reports pointed out that the Wnt/*β*-catenin signaling pathway take part in the advance of breast cancer, which indicated the poor prognosis of TNBC associated with the abundance of the Wnt/*β*-catenin pathway [5–7, 19]. Therefore, with tunicamycin treatment, the viability and apoptosis-related molecular protein Bcl-2 and Bax expression both reduced due to the Wnt/*β*-catenin pathway was inhibited and clearly induced by tunicamycin (Figures 1(c) and 1(d)). Therefore, we hypothesized that tunicamycin could induce cell apoptosis via the repress of the Wnt/*β*-catenin pathway.

In order to identify whether tunicamycin-induced ER stress can block the Wnt/*β*-catenin pathway, Licl was delivered to cells combined with tunicamycin. From Figure 2(a), we can see that LiCl successfully counteracted the inhibition effect of tunicamycin-activated Wnt/*β*-catenin pathway again. Furthermore, the Bax and Bcl-2 expression and AO/EB staining revealed that the cell apoptosis was suppressed by the initiation of *β*-catenin pathway (Figures 3(a) and 3(b)). Indeed, deposition of *β*-catenin transferred from cytoplasm to the nucleus and activated the transcription genes mediated by T-cell factor/lymphoid enhancer factor (TCF/LEF) related to the formation of breast tumor [20, 21]. However, as the downstream gene of the Wnt/*β*-catenin signaling pathway, c-Myc affects the tumor cell cycle by inhibiting growth suppression gene transcription and was significantly increased in Tun + Li group compared with Tun treatment (Figure 3(c)), which could lead to poor survival and continuous growing of MDA-MB-231 cells [22]. Recently, Xu et al. also found similar experiment results and investigated the possibility that Schisandrin A could suppress the cell cycle and introduce apoptosis of cells in TNBC though the Wnt/ER stress signaling pathway. However, they merely researched the activation of the Wnt/*β*-catenin and ER stress-related protein expression [23]. Collectively, our study confirmed the specific progress of the pathway in that cell apoptosis was induced by ER stress through suppressing the Wnt signaling pathway by combination delivery with tunicamycin and LiCl (Figure 4).

Although the study lacks a contrasting experiment between different cell lines of breast cancer and animal experiment, it firstly and sufficiently verified the relationship between the Wnt/*β*-catenin pathway and endoplasmic reticulum stress in TNBC. Thus, further research should be conducted on the project of in vivo experiment and the verification of mechanism in different cell lines. Collectively, this study inspected the specific mechanism that the *β*-catenin signaling pathway affected the apoptosis process which was introduced by ER stress in MDA-MB-231 cells, which proved a potential treatment target and reduction of side effects.

## 5. Conclusions

This study investigated whether activation of ER stress by tunicamycin could induce apoptosis of TNBC in MDA-MB-231 cells. The processes were initiated through repressing the Wnt/*β*-catenin signaling pathway, which could be reversed by LiCl (Figure 4). In conclusion, all of our data inspected the specific mechanism of the apoptosis initiated by ER stress and provided a theoretical basis for further research and treatment.

## Figures and Tables

**Figure 1:** Tunicamycin induces apoptosis in MDA-MB-231 cells and its Wnt/*β*-catenin pathway in a dose-dependent manner. Different doses of tunicamycin were used to treat the MDA-MB-231 cells. (a–c) Western blotting shows the level of GRP78, CHOP, *β*-catenin, phospho-*β*-catenin, and apoptosis proteins, Bcl-2 and Bax. Three independent experiments were performed. (d) Cell viability was measured by an MTT assay. Six independent experiments were performed. Values shown (*n* = 3 or 6) are the mean ± SD, ^*∗*^*P* < 0.05 or ^*∗∗*^*P* < 0.01 compared with 0 group.

**Figure 2:** *β*-catenin pathway is inhibited by endoplasmic reticulum (ER) stress. (a) Western blotting shows the decreased *β*-catenin level and the increased phospho-*β*-catenin level. (b) The expression of GRP78 and CHOP was determined using western blot. Three independent experiments were performed, and GAPDH was used as the internal control. Values shown (*n* = 3) are the mean ± SD, ^*∗*^*P* < 0.05 or ^*∗∗*^*P* < 0.01 compared with the control group; ^#^*P* < 0.05 or ^##^*P* < 0.01 compared with Tun + Li. C group of MDA-MB-231 cells cultured normally with no treatment; Tun groups were delivered with tunicamycin; Li groups were delivered with LiCl; Tun + Li groups were delivered with tunicamycin and LiCl.

**Figure 3:** Tunicamycin inhibits the Wnt/*β*-catenin signaling pathway to affect the viability of MDA-MB-231 cells. (a) Western blotting show the relative level of apoptosis-related proteins, Bax and Bcl-2, upon various treatments of tunicamycin and LiCl. Three independent experiments were performed, and GAPDH was used as the internal control. (b) The apoptosis in MDA-MB-231 cells was measured using acridine orange/ethidium bromide (AO/EB) staining. (c) The expression of c-Myc was measured using western blot. Three independent experiments were performed, and GAPDH was used as the internal control. Values shown (*n* = 3) are the mean ± SD, ^*∗*^*P* < 0.05 or ^*∗∗*^*P* < 0.01 versus the control group; ^#^*P* < 0.05 or ^##^*P* < 0.01 compared with Tun + Li group. C group of MDA-MB-231 cells was cultured normally with no treatment; Tun groups were delivered with tunicamycin; Li groups were delivered with LiCl; Tun + Li groups were delivered with tunicamycin and LiCl.

**Figure 4:** Mechanism of tunicamycin-induced ER stress promotes breast cancer cell MDA-MB-231 apoptosis. Tunicamycin is an activator of ER stress. It inhibits the ER glycosylation process and causes ER stress. After ER stress is activated, it inhibits the Wnt signaling pathway. When this pathway is suppressed, *β*-catenin phosphorylation is increased, resulting in a decrease in nuclear *β*-catenin, affecting the activation of downstream gene c-Myc transcription, and ultimately promoting breast cancer cell MDA-MB-231 apoptosis.

## Data Availability

The data used to support the findings of the study have not been made available because analytical permission was not obtained from the data provider.
